# The Method of Reconstructing Three-Dimensional Human Posture from Two-Dimensional Images in Film and Television Production

**DOI:** 10.1155/2022/2419123

**Published:** 2022-07-06

**Authors:** Yuanyuan Zhao, Jiexiao Tang

**Affiliations:** College of Art and Media, Hefei Normal University, Hefei, Anhui 230601, China

## Abstract

With the development of computer software and hardware technology, film and television production has made a breakthrough. More and more film and television works have changed from the traditional plane two-dimensional space projection to three-dimensional space projection. Three-dimensional works give the audience an immersive feeling. Taking human posture, one of the most important components in film and television works, as an example, this paper discusses the method of reconstructing three-dimensional human posture from two-dimensional images in film and television production. Starting from the research significance of two-dimensional image reconstruction of three-dimensional human posture in film and television production, the existing three-dimensional human posture in film and television production is analyzed. The audience can watch the film and television works in an all-round way to keep the film and television works fresh to the greatest extent. This paper provides a certain reference value for 3D stereoscopic projection.

## 1. Introduction

From the perspective of film and television production methods, two-dimensional film and television production is to create each picture directly through plane drawing and then make film and television works. In 3D film and television production, the draft layout of the image to be created is usually carried out in the two-dimensional plane, then the three-dimensional modeling is carried out through computer technology, and finally the final film and television effect is made through rendering and other actions [1]. Therefore, from the perspective of picture expression, since the two-dimensional creation method can be completed only through drawing, the expression method of two-dimensionalimage is freer, and various deformation effects can be easily achieved through drawing pictures. 3D creation requires 3D modeling. Therefore, in order to avoid the loss of time, energy, and cost caused by frequent model modification, except for special modeling when special perspective picture is required, deformation rarely occurs in 3D animation picture [2]. Therefore, in two-dimensional film and television works, we can more frequently see very exaggerated forms of expression, such as the exaggerated drawing of people's facial expression in different scenes, the O-shaped mouth when surprised, the drawing of a line around the eyes when expressing the character's silent mood, and so on. These expressions add three-dimensional unrealized vitality to two-dimensional animation. On the other hand, it is precisely because 3D film and television works need to be modeled. Although this process leads to less changes in character modeling, it lacks the expressive vitality of 2D works. However, it is for this reason that the expressiveness of three-dimensional is relatively stable, and all performances are determined by the model, which is minimally affected by the painter [3]. For example, two-dimensional film and television works often encounter the problem of unstable work quality due to the change of painters or other environmental factors. In terms of production cycle, Ovi film and television does not need complex computer operations, such as model production, scene layout, material, and lighting [4]. Therefore, the time and capital of two-dimensional film and television are mainly spent on the manual drawing of each frame. The focus of 3D film and television is on the process links required for model production, scene layout, and material. However, when the early model and corresponding preparation links are determined, the remaining specific production actions can be carried out by the computer according to the program compiled in advance [5]. Although in the way of film and television production, picture expressiveness, and production cycle, two-dimensional film and television and three-dimensional film and television have different characteristics. However, due to the limitations of the basic creation method of two-dimensional animation, hand drawing, it is difficult to show the perspective effect in the scene and viewing angle. Therefore, perspective painters generally choose to express the perspective effect through the perspective angle of the character. The performance of the scene is mainly carried out through rich color levels, which leads to the fact that in order to avoid color conflict with the scene, the protagonist's color levels are usually only light and dark [6]. 3D film and television can automatically calculate the perspective scene effect change through the computer parameters set in advance, so the perspective level effect change and color change of characters and scenes are very rich. At the same time, during the application of 3D film and television in the scene, different scene materials can be realized through different plug-ins, which makes the picture texture of 3D film and television more intense, which is impossible for 2D film and television [7].

Taking human posture, one of the most important components in film and television works, as an example, this paper discusses the method of reconstructing three-dimensionalhuman posture from two-dimensional images in film and television production. The innovation of this paper is to modify the 3D reconstruction process of some joints that have a significant impact on human posture in the current algorithm. To solve the problem of insufficient two-dimensional image data sets, the neural network algorithm is used to optimize the iterative calculation, which greatly improves the speed of three-dimensional human posture reconstruction.

## 2. Related Work

At present, the commonly used three-dimensional human pose reconstruction technology is mainly divided into three categories according to the different generation methods of the reconstructed model. The first is to generate the three-dimensional human pose model through the three-dimensional human body scanning equipment. The second is to generate the reconstructed three-dimensional human pose model based on the existing human body database. The third is based on two-dimensional data generated by spatial color images [8]. The first method is based on 3D human body scanning equipment for 3D human body pose reconstruction. Because the 3D human body scanning equipment used is expensive and the operation is relatively professional, professional personnel are needed for debugging. Therefore, although the equipment has high accuracy and high accuracy, it is not suitable for being widely used in the film and television industry [9]. At present, the equipment is only used in scientific experiments. For example, Yang et al. scan the research object through the three-dimensionalhuman body scanning equipment as well as record the corresponding three-dimensional coordinates in the scanning process and turn them into corresponding data files. After preprocessing the data, the three-dimensional human body pose model of the target object is generated according to the key points [10]. The second method, the reconstruction of 3D human pose model based on human body part database, belongs to the method of 3D human pose generation in earlier times. This method mainly depends on the data of posture of various parts of the human body collected in the database. Users first determine the data they need before use and then screen it in the database to generate the required three-dimensional human posture model. Huang et al. obtained the three-dimensional model of the target human posture by using the three-dimensional model data of various human postures in human pose modeling software database. By studying and combining the data of different three-dimensional human pose databases, Li et al. proposed a new three-dimensional human model generation engine. The algorithm can automatically generate the corresponding three-dimensional human pose model through the two-dimensional images from different angles and relevant human pose data provided by the user [11].

Due to the limitations of the first two three-dimensional human pose reconstruction methods, the current common application is to reconstruct the three-dimensional human pose model based on two-dimensional images. This method mainly locates the preliminary data information through the two-dimensional color image of the target object, then transforms the data into human posture data in three-dimensional space through a specific two-dimensional to three-dimensional deformation standard three-dimensional human body template, and finally generates a three-dimensionalmodel with the same human posture as that in the two-dimensional color image. This method has the advantages of simple data source, simple operation, and low cost and avoids the influence of the particularity of database data on the reconstruction results. Therefore, it has become the mainstream method of two-dimensional image reconstruction of three-dimensional human posture in film and television production [12]. Lin et al. first proposed the method of reconstructing three-dimensional human posture model through two two-dimensional color images of human body front view and side view. Based on this, Ji et al.'s further research found that two-dimensional orthogonal contours can be generated from two two-dimensional images, and the accuracy of the reconstructed three-dimensional human posture can be further improved based on the method of depth learning. Zhu et al. explored the influence of different clothes on the reconstruction of three-dimensional human posture and summarized how to accurately grasp the characteristics of three-dimensional human posture reconstruction through two-dimensional images when wearing ordinary or loose clothes [13]. To solve the problem of how to create a three-dimensional human pose model when there is only a two-dimensional color image of a single human eye body, Mathew et al. first proposed a parametric standard three-dimensional human pose template SMPL, which is similar to the method of reconstructing a three-dimensional human pose model through a database. Users can filter and automatically generate the corresponding three-dimensional human pose model only through the data extracted from a single photo of the target human body [14]. In addition to the above three-dimensional human model reconstruction methods, Zhao et al. have developed other methods, such as data-driven method, reconstruction method based on target human video, personalized human editing method, and so on, which also have their own advantages and disadvantages. Due to the length of this article, I will not repeat it here [15].

## 3. Method

At present, in the algorithm of reconstructing three-dimensional human posture from two-dimensional images, the changes of joint points in the reconstruction process are often ignored, which leads to abnormal problems in the reconstructed three-dimensional human posture, violates the basic physiological structure of the human body, and causes some bad visual feelings to the audience. The main factors affecting the posture of human body are the elbow and knee joints of human body. When the human body presents different states, such as curling, stretching, or grasping, there will be different changes in the muscle stretching degree, joint orientation, joint concave convex state, and so on of the corresponding elbow and knee joints. This paper modifies the three-dimensional reconstruction process of some joints that have a significant impact on human posture in the current algorithm. In view of the lack of data set of two-dimensional images, the optimization iterative calculation is carried out through neural network algorithm, which greatly increases the speed of reconstructing three-dimensional human posture from two-dimensional images. The specific research framework is shown in Figure 1.

In the research field of two-dimensional image reconstruction of three-dimensional human posture, because different human posture is also different in the process of three-dimensional reconstruction, we usually divide human posture into two categories. One is the stretching posture, such as our common a posture (feet naturally separated, hands naturally extended downward on both sides of the body), and t posture (feet naturally separated, hands on both sides of the body and parallel to the ground), as well as some other stretching postures. These poses are usually very close to the zero pose of the human body template. Therefore, when the two-dimensional image of the target human body is called the extended pose, the reconstruction of the three-dimensional human body pose is usually less difficult. The other is nonstretching posture, which is mostly irregular. Due to the needs of the film and television field, it may also be some specific postures or actions. At this time, the joints of the main human body are in an unnatural state, which makes it difficult to extract the data correctly. It also leads to the inaccuracy of extracting the joint point data in the two-dimensional image when reconstructing the three-dimensionalhuman posture, Furthermore, the posture of three-dimensional human body does not accord with the physiological structure of human body. Human skeleton extraction is a very important research direction in the field of computer vision. With the increasing improvement of computer hardware and the exponential enhancement of computing power, great progress has been made in image processing. Therefore, the demand for processing and analyzing human movements on the computer is also increasing. Human skeleton extraction technology is the basis of analyzing behavior, which has very important practical value. Therefore, this paper proposes the idea of iterative fitting optimization to extract the human joint point information from the human posture in the two-dimensional image from the bottom-up and mainly calculate the distance between the relevant nodes in the two-dimensional image through the triangle similarity principle, as shown in the following formula.

(1) $$\begin{array}{c} \frac{Fc}{Li}=\frac{Lcm}{Lm}. \end{array}$$

The calculation premise is that the formula is valid when the target human body is parallel to the image plane. Therefore, when the premise that the target human body is parallel to the image plane is not satisfied, we need to obtain the optimal solution of the global orientation of the human body through calculation. See the following formula for specific objective function.

(2) $$\begin{array}{c} E\left(\beta ,\theta \right)=E_{j}\left(\beta ,\theta ,K,J_{est}\right)=\sum_{ji}\varpi_{i}\rho \left(\prod_{k}\left(R_{\theta }\left(J{\left(\beta \right)}_{i}\right)\right)-J_{est}\right). \end{array}$$

However, in the specific operation, we found that this method will bring great errors and even lead to the problem of key orientation errors in the subsequent three-dimensional reconstruction of human posture. Therefore, we can reduce the error by changing different penalty terms in the objective function. The specific penalty term expression is shown in the following formula.

(3) $$\begin{array}{c} E_{\theta }\left(\theta \right)=\underset{j}{\min}\left(-\log\left(cg_{i}N\left(\theta ;u_{\theta ,j},\sum \theta ,j\right)\right)\right). \end{array}$$

The error of joint points is significantly reduced after adding the penalty error, and the change of error value before and after adjustment is shown in Figure 2.

From Figure 2, we can see that the reconstruction error value of each key point is reduced by adjusting the penalty term. The error values of each part are different, in which the error reduction value of the upper limb elbow joint is about 25, while the error value of the knee joint is about 23. Overall, the reduction range of the error value of the lower limb joint is significantly higher than that of the upper limb joint. Through the front and rear data, we preliminarily speculate that the accuracy of the previous algorithm for the lower limb joint points is lower than that of the upper limb joint points. Therefore, after the algorithm is adjusted, the reconstruction frequency of joint points of upper and lower limbs is adjusted to the same level. At this moment, because the accuracy level of lower limb joint points before adjustment is low, the optimization range of error value after adjustment is large. However, overall, the reconstruction errors of the adjusted joint points decreased, and the reconstruction accuracy increased.

After determining the selection of joint points, we continue to extract the position of human skeleton from top to bottom through DeepCut algorithm. DeepCut algorithm runs based on neural network. It first obtains the approximate candidate body parts through the determined position of joint points. In human physiological structure, each joint point is connected with a part of the body, so the position of the joint point can roughly obtain the body part. This creates a dense map of the reconstructed target body. This figure is similar to the general structure of neural network. There is a certain correlation between different points, and the correlation between joint points with close physiological structure is large (e.g., the joint point between tibia and fibula is the key point to jointly determine the leg posture due to up and down effects). On the contrary, the correlation is relatively small. Next, the position extraction of the whole human skeleton can be regarded as an optimization problem based on neural network algorithm. The specific expression is shown in the following formula.

(4) $$\begin{array}{c} f^{\prime }\left(x_{k-1}\right)=\frac{f\left(x_{k-1}\right)}{x_{k-1}-x_{k}}. \end{array}$$

The expression of *X* can be obtained by Fourier transform. See the following formula for details.

(5) $$\begin{array}{c} x_{k}=x_{k-1}=\frac{f\left(x_{k-1}\right)}{f^{\prime }\left(x_{k-1}\right)}. \end{array}$$

When the *k*th independent variable is infinitely close to the *k* − 1 independent variable, the function root can be obtained. At this moment, the function expression is shown as follows.

(6) $$\begin{array}{c} x_{k}=x_{k-1}=\frac{f^{\prime }\left(x_{k-1}\right)}{f^{\prime \prime }\left(x_{k-1}\right)}. \end{array}$$

The algorithm is based on SMPLify model, but the three-dimensional human posture model reconstructed by this algorithm generally has the problem of natural bending of joints, so we improve the algorithm. By adding a priori term of pose, the key points of the constructed three-dimensional human pose model can be predicted in advance through the two-dimensional image. The specific expression of attitude a priori term is shown as follows.

(7) $$\begin{array}{c} m_{k}\left(s\right)=f_{k}+g_{k}^{T}s+\frac{1}{2}s^{T}G^{k}s. \end{array}$$

On this basis, we further supervise the reconstruction process of 3D human pose model through matrix. The matrix expression is shown as follows.

(8) $$\begin{array}{c} R\left(\alpha ,\beta ,\gamma \right)=R_{z}\left(\alpha \right)R_{y}\left(\beta \right)R_{x}\left(\gamma \right). \end{array}$$

Finally, we named the optimized algorithm SMPLify-m and used SMPLify algorithm and SMPLify-m algorithm to reconstruct the three-dimensional human pose model of the target object. In order to eliminate the influence of irrelevant variables, we select the two-dimensional image of the same reconstruction object for preparation. The results are shown in Figure 3.

Figure 3 is the result of three-dimensional human pose model reconstruction through two-dimensional color images taken in the front and left directions of the target object. The abscissa is the overall global orientation of the target object's body, and the ordinate represents the bending angle value of the corresponding joint position. It can be seen that, for the reconstruction of elbow joint, the joint bending reconstructed by SMPLify algorithm decreases first and then increases with the increase of the overall orientation of the target. In the three-dimensional human posture model reconstructed by SMPLify-m algorithm proposed in this paper, the bending degree of elbow joint increases first and then decreases with the increase of the overall orientation of human body. By comparing with the actual situation, we can see that the SMPLify proposed in this paper is more in line with the physiological change law of human body. For the knee joint, the overall change trend is not so clear compared with the elbow joint, but there is a great difference in the change trend of knee joint bending angle calculated by SMPLify and SMPLify-m algorithm. For SMPLify algorithm, there is no great change in knee joint bending angle as a whole; only there is a large fluctuation near the positive direction, and the bending degree increases. The knee joint curvature obtained by SMPLify-m is opposite to the former, and there is a large fluctuation on both sides of 0. In fact, when our body is facing nonforward, the corresponding knee joint will bend to a certain extent. Therefore, it can be determined that the 3D human posture reconstructed by SMPLify-m algorithm proposed in this paper is more in line with the characteristics of human physiological structure.

After determining the algorithm of two-dimensional image reconstruction of three-dimensional human posture, considering that the production cycle of two-dimensional image reconstruction of three-dimensional model in film and television production mainly takes a long time in the early stage, this paper hopes to improve the efficiency of two-dimensional image reconstruction of three-dimensional human posture. In the production process of traditional algorithms, the whole process is usually rendered through the optimization iteration algorithm, and the optimization iteration is carried out under the random walking mechanism. See the following formula for the specific expression.

(9) $$\begin{array}{c} x_{i}^{\prime }=x_{i}+Rand\left(-\varepsilon ,\varepsilon \right),i=1,2,\ldots ,N. \end{array}$$

There are different probability events in the random process. Generally, in the optimization process, we use the probability function to calculate the corresponding probability value. See the following formula for details.

(10) $$\begin{array}{c} P\left(X,X^{\left(new\right)}\right)=\left\{\begin{array}{cc} 1, & F\left(X^{new}\right)<F\left(X\right)\\ e^{\frac{\Delta F}{\lambda }}, & other \end{array}\right... \end{array}$$

In the calculation process, we need to ensure the minimum residual. At this time, the function value is the optimal solution. Thirdly, we optimize through the quaternion algorithm to ensure the minimum residual.

(11) $$\begin{array}{c} \left\|q\right\|=\sqrt{qq^{\prime \prime }}=\sqrt{q_{0}^{2}+q_{1}^{2}+q_{2}^{2}+q_{3}^{2}}. \end{array}$$

When the orientation angle of the target object changes, taking the center of gravity of the target object as the origin, the quaternion representation on each coordinate axis is shown in formulas (12) to (14).

(12) $$\begin{array}{c} q_{x}=\left[\cos\frac{\phi }{2},\left(\sin\frac{\phi }{2},0,0\right)\right], \end{array}$$

(13) $$\begin{array}{c} q_{y}=\left[\cos\frac{\theta }{2},\left(0,\;\sin\frac{\theta }{2},0\right)\right], \end{array}$$

(14) $$\begin{array}{c} q_{z}=\left[\cos\frac{\psi }{2},\left(0,0,\;\sin\frac{\psi }{2}\right)\right]. \end{array}$$

The Euler angle is expressed as follows.

(15) $$\begin{array}{c} \left[\begin{array}{c} \phi \\ \theta \\ \psi \end{array}\right]=\left[\begin{array}{c} a\;\tan\frac{2\left(q_{0}q_{1}+q_{2}q_{3}\right)}{1-2\left(q_{1}^{2}+q_{2}^{2}\right)}\\ a\;\sin\left(2\left(q_{0}q_{2}+q_{1}q_{3}\right)\right)\\ a\;\tan\frac{2\left(q_{0}q_{3}+q_{1}q_{2}\right)}{1-2\left(q_{2}^{2}+q_{3}^{2}\right)} \end{array}\right]. \end{array}$$

Because the algorithm is trained end to end and has the powerful graphics computing ability of convolutional neural network, we named the algorithm hmr-SMPLify-x algorithm. By continuously adjusting SMPL-x parameters, the algorithm obtains the optimal solution of the function when the error function gradually converges. The specific training process is shown in Figure 4.

In the training process, we set the training times as 700 epochs, the activation function as Adam function, and batch_Set the size to 32. Under this condition, the mean square error of 185 parameters under the three-dimensional human posture model is calculated. As can be seen from Figure 4, with the increase of training times of convolutional neural network, the error value gradually decreases and finally converges and tends to balance. There are also some fluctuations in the middle. We speculate that the small area fluctuation caused by the initial value is still decreasing as a whole. In addition, we have compared the randomization. The results show that compared with the random error, the error calculated by the hmr-SMPLify-x algorithm proposed in this paper is significantly lower than that of randomization, which shows that the overall performance of the two-dimensional image reconstruction three-dimensional human posture model algorithm proposed in this paper is better.

## 4. Result Analysis and Discussion

Through the above research, we can get that the most commonly used three-dimensional human posture method is two-dimensional image reconstruction. In the traditional two-dimensional image reconstruction method of three-dimensional human pose, the corresponding morphological data will be obtained from the two-dimensional image of the target reconstruction object, and then the three-dimensional human pose model will be generated by comparing the three-dimensional human template deformation standard. At the same time, according to different data sources, it can be divided into the method of generating and reconstructing three-dimensional human posture model from multiple two-dimensional color images (i.e., more than two) and the method of reconstructing three-dimensional human posture from a single two-dimensional color image, as shown in Figure 5.

However, either method is based on the iterative fitting optimization algorithm. By constantly adjusting the parameters and changing the key data information affecting the human body posture, the accurate three-dimensional human body posture data can be found when the plane projection of the reconstructed three-dimensional human body posture corresponds to the posture key points on the two-dimensional image of the data source. However, because the changes of joint activities under different postures of human body in three-dimensional state have certain physiological characteristics, the joint point states under different postures have subtle differences in physiological structure. Finally, we take Figure 5 as an example to verify the accuracy and speed of 3D reconstruction of SMPLify-m algorithm and SMPLify-x algorithm proposed in this paper.

Firstly, we compare the difference between the previous algorithms and the SMPLify-m algorithm proposed in this paper in the accuracy of two-dimensional image reconstruction of three-dimensional human posture, as shown in Figure 6.

Figure 6 shows the evaluation results of the accuracy of reconstructing 3D human posture based on 2D images through different algorithms. The abscissa represents the type of algorithm and the ordinate represents the accuracy of the algorithm. Since the dense correspondence between 2D RGB image and 3D stereo model is to be established, a traditional method is to find a point on the image and then rotate the image and stereo model to achieve accurate coordinate positioning, but the efficiency is too low. Therefore, they divided the marking work into two stages: first, the macro part segmentation and then, the specific corresponding annotation. The evaluation is mainly carried out from two dimensions: the whole-body contour and partial hierarchical contour of the target object. On the whole, the accuracy of the algorithm based on the whole-body contour pose is higher than that of the partial hierarchical contour pose. We speculate that this is due to the data acquisition of the two-dimensional whole-body image in the standard algorithm model, so it may be inaccurate when inferring the partial contour pose based on this. In addition, it can be seen that the reconstruction accuracy of the existing common algorithms for the whole-body contour and posture is maintained at about 92%, but the reconstruction accuracy of the SMPLify-m algorithm proposed in this paper is about 95%.

Next, we monitor the operation efficiency of the algorithm in this paper. Still taking Figure 5 as an example, we calculate the time required to reconstruct the three-dimensionalhuman posture model from the two-dimensional image under different algorithms. The specific results are shown in Figure 7.

In the reconstruction process, we select the expose dataset as the reference template for 3D reconstruction, and the operating system used in the experiment is Ubuntu 16.04. From Figure 7, we can see that the total time difference of existing algorithms in reconstructing three-dimensional human posture model based on two-dimensional image is small, but the average time is different. The hmr-SMPLify-x algorithm proposed in this paper takes the lowest time in the reconstruction process, and the average time is also the lowest.

## 5. Conclusion

Starting from the research significance of image reconstruction in film and television production, this paper analyzes the existing two-dimensional image reconstruction methods of three-dimensional human posture in film and television production and puts forward its own views on its shortcomings. Taking human posture, one of the most important components in film and television works, as an example, this paper discusses the method of reconstructing three-dimensional human posture from two-dimensional images in film and television production. Taking human posture, one of the most important components in film and television works, as an example, this paper discusses the method of reconstructing three-dimensional human posture from two-dimensional images in film and television production. The innovation of the research lies in modifying the three-dimensional reconstruction process of some joints that have an important impact on human posture in the current algorithm. Aiming at the shortage of two-dimensional image data sets, neural network algorithm is used to optimize the iterative calculation, which greatly improves the speed of three-dimensional human posture reconstruction.

## Figures and Tables

**Figure 1:** Reconstruction of 3D human body model from 2D color image based on iterative fitting optimization.

**Figure 2:** The algorithm adjusts the reconstruction error values of the front and rear nodes.

**Figure 3:** Comparison of the effect of two-dimensional color image reconstruction of three-dimensional human pose model.

**Figure 4:** Convolutional neural network module training process curve.

**Figure 5:** Two-dimensional image of the target body.

**Figure 6:** Evaluation results of reconstruction accuracy algorithm based on whole-body contour and partial classification.

**Figure 7:** Different algorithms reconstruct speeds on expose data sets.

## Data Availability

The data used to support the findings of this study are available from the corresponding author upon request.
